# Using Patient-Derived Xenografts to Explore the Efficacy of Treating Head-and-Neck Squamous Cell Carcinoma With Anlotinib

**DOI:** 10.3389/pore.2021.1610008

**Published:** 2021-12-09

**Authors:** Fangling Hu, Liang Guo, Jieqing Yu, Daofeng Dai, Yuanping Xiong, Yuanqiao He, Wensheng Zhou

**Affiliations:** ^1^ Department of Otolaryngology-Head and Neck Surgery, First Affiliated Hospital of Nangchang University, Nanchang, China; ^2^ Jiangxi Institute of Otorhinolaryngology-Head and Neck Surgery, Nanchang, China; ^3^ Laboratory Animal Science Center of Nanchang University, Nanchang, China

**Keywords:** head-and-neck squamous cell carcinoma, drug sensitivity, patient-derived xenograft, anlotinib, tumor inhibition

## Abstract

**Objective:** The efficacy of anlotinib as a treatment for head-and-neck squamous cell carcinoma (HNSCC) has been little explored. Here, we used patient-derived xenografts (PDXs) to this end.

**Methods:** Fresh tumor tissues of HNSCC patients were screened in terms of *in vitro* drug sensitivity using the MTT assay. Patient PDXs were used to confirm the anti-tumor effects of anlotinib *in vivo*. After the medication regimen was complete, the tumor volume changes in mice were calculated. Apoptosis was measured using the TUNEL assay. The cell proliferation and apoptosis levels of PDXs yielded data on the utility of anlotinib treatment *in vivo*.

**Results:** Anlotinib suppressed the *in vitro* proliferation of nine tumor tissues by an average of 51.05 ± 13.74%. Anlotinib also significantly inhibited the growth of three PDXs in mice (tumor growth inhibition 79.02%). The expression levels of Ki-67 and proliferating cell nuclear antigen after anlotinib treatment were significantly lower than those in the controls. The negative and positive controls exhibited no and some apoptosis, respectively, whereas the anlotinib group evidenced extensive apoptosis.

**Conclusion:** Anlotinib suppressed HNSCC growth *in vitro* and *in vivo* (by inhibiting cell proliferation and promoting apoptosis), suggesting that anlotinib can potentially treat HNSCC.

## Introduction

Head-and-neck cancers arise from the mucosal surfaces of the oral and sinonasal cavities, oropharynx, hypopharynx, and larynx. Such cancers constitute the seventh most common cancer group worldwide (3% of all malignancies in 2018) (1). Over 90% of such cancers are head-and-neck squamous cell carcinomas (HNSCCs), with over 890,000 new cases and 450,000 deaths reported annually in the United States (1, 2). There are several risk factors, of which smoking and alcohol consumption are the most common (3, 4). Recently, human papillomavirus has been confirmed to contribute to oropharyngeal carcinoma development, especially in young males (5). Although surgery, radiation therapy, chemotherapy, and combination therapy have been used to treat HNSCC for decades, the prognosis remains unsatisfactory (6, 7).

Angiogenesis plays a key role in the creation, development, and metastasis of solid tumors. Therefore, anti-tumor angiogenesis therapies have become popular. Vascular endothelial growth factor (VEGF) is key in terms of tumor angiogenesis. VEGF triggers downstream signaling by activating three structurally related VEGF receptor (VEGFR) tyrosine kinases (VEGFR1, VEGFR2, and VEGFR3), thus promoting tumor angiogenesis and metastasis (8–13).

Anlotinib is a very potent, multi-targeting, oral tyrosine kinase inhibitor that blocks VEGFR2 phosphorylation as well as the actions of platelet-derived growth factor receptor α/β (PDGFR α/β), c-Kit, Ret, Aurora-B, c-FMS, and the discoid region of domain receptor 1 (DDR1) (14, 15). Anlotinib also inhibits tumor angiogenesis induced by VEGF, PDGF, and FGF-2 (16, 17). Phase II/III clinical trials revealed that anlotinib had encouraging effects in patients with a variety of solid tumors, including non-small‐cell lung cancers, hepatocarcinomas, renal carcinomas, gastric cancers, and soft tissue sarcomas (15). The efficacy of anlotinib in patients with advanced lung squamous cell carcinomas has been confirmed in clinical trials, and the drug is approved as the third-line treatment for such cancers (18). We hypothesized that anlotinib would inhibit HNSCC growth, invasion, and metastasis and would usefully treat refractory advanced cancers. As no report on the potential anti-tumor effects of anlotinib on animal HNSCC has appeared, we collected fresh HNSCC samples and constructed patient-derived xenografts (PDXs) to explore the therapeutic effects of the drug.

## Materials and Methods

### *In Vitro* Drug Sensitivities

All samples were collected at the First Affiliated Hospital of Nanchang University and all procedures were approved by the ethics committee of the hospital (approval no. 017). Informed patient consent was obtained before surgery. Nine HNSCCs were surgically removed, divided into 2 × 2 × 2 mm^3^ sections, and placed in 96-well plates (one block/well) at a low temperature. After injection of a water-containing gel, the tissues were cultured at 37°C at 95% humidity under 5% (v/v) CO_2_. Three-quarters of the medium containing different drugs was changed every 1–2 days. The control cells were treated with Dulbecco’s modified Eagle medium/F12 complete medium (Cat. No.11330107; Gibco, Amarillo, TX, United States) supplemented with 10% (v/v) fetal bovine serum (Cat. No.16140063; Gibco), 100 units/ml penicillin, and 100 μg/ml streptomycin. The tissues in the control groups were cultured in a manner similar to control cells. The drug groups were cultured in complete medium with 3% (v/v) dimethyl sulfoxide (DMSO, Cat. No. D4540; Sigma, St. Louis, MO, United States), 24 µM anlotinib (Zhengda Tianqing Pharmaceutical Group Co. Ltd., Nanjing, China), 20 µM sunitinib (Pfizer Pharmaceuticals Ltd., New York, NY, United States), 9 µM apatinib (Hengrui Pharmaceuticals, Jiangsu, China), 75 μg/ml paclitaxel (Beijing SL Pharmaceutical Co. Ltd., Beijing, China), or 25 μg/L cisplatin (Harvey, United States). The culture medium was replaced after 24 h to maintain the activity and morphology of the original tissue block. On day 8, the medium was removed, tissues were washed three times with phosphate-buffered saline, and MTT solution (Sigma) was added. After incubation for 16 h, the tissue blocks were placed in new 96-well plates, and each block was incubated with 200 µl DMSO for 6 h. Aliquots of 100 µl DMSO were then placed into the wells of a fresh 96-well plate, and the absorbance (A values) at 490 nm were measured. Drug sensitivity was assessed based on the tumor inhibition rate, which was calculated as [1—(drug A-blank A/control A-blank A)] × 100%; a tumor inhibition rate ≥30% was presumed to indicate drug sensitivity. The experiment was repeated three times and averages were calculated.

### PDXs

PDXs (numbered as P0) were established. Three PDX models, one of hypopharyngeal carcinoma and two of laryngeal carcinomas, were selected and passaged to P3 by the same method, then used for *in vivo* experiments. When the diameters of the third-generation subcutaneous tumors reached 1 cm, they were minced (2 × 2 × 2 mm^3^) and subcutaneously implanted into the flanks of 4- to 6-week-old nude mice. Each PDX was inoculated into 24 mice. When the tumor volumes reached 100–200 mm^3^, the mice were randomly divided into three groups of six: a control group (normal saline 100 μl intragastrically per day), a drug group (anlotinib 3 mg/kg intragastrically per day), and a positive control group (cisplatin 5 mg/kg intraperitoneally per week). Mouse health and tumor growth were observed daily. The tumor volume and mouse body weight were recorded every 4 days. Twenty-one days later, when the tumor volume in the control group reached 1,500 mm^3^, all mice were sacrificed via cervical dislocation, and the tumor tissues were harvested. Tumor size was measured using a caliper, and tumor volume was calculated as 1/2 × length × (width)^2^. Tumor growth inhibition (TGI) was used to evaluate the anti-tumor effects of anlotinib. TGI (%) was calculated as: TGI (%) = [1—(tumor volume at the end of the drug treatment group—tumor volume at the beginning of the drug treatment group)/(tumor volume at the end of the control group—tumor volume at the beginning of the control group)] × 100%. All experiments were approved by the Animal Ethics Committee of Nanchang Leyou Biotechnology Co. Ltd.

PDX construction was performed using the protocol established by Karamboulas et al. (19). Briefly, HNSCC-PDXs were generated, the tumor tissues were processed, and the PDX models were expanded into cohorts for drug testing.

### Pathology

Formalin-fixed PDX samples were embedded in paraffin and cut into 3-µm-thick sections that were baked at 60°C for 12 h. The sections were then placed into xylene for 5–10 min (repeated three times), hydrated in 100, 100, 95, 85, and 75% (w/w) ethanol (in sequence) for 5 min each, soaked in distilled water for 5 min, stained with hematoxylin (Wellbio, China) for 5–10 min, washed with distilled water, stained with eosin (Wellbio) for 3–5 min, washed with distilled water, dehydrated in 95 and 100% (v/v) alcohol baths for 5 min each, placed in xylene for 10 min (two repeats), mounted with neutral gum, and observed microscopically.

### Terminal Deoxynucleotidyl Transferase-Mediated Deoxyuridine Triphosphate Nick-End Labeling Immunohistochemistry

After dewaxing, some tissues were used for immunohistochemistry and TUNEL assays. Some slides were subjected to Proteinase K incubation and used for permeabilization; positive slides were incubated with recombinant terminal deoxynucleotidyl transferase enzyme, Equilibration Buffer, dUTP Labeling Mix, whereas negative slides were incubated with distilled water instead of recombinant terminal deoxynucleotidyl transferase enzyme. The TUNEL Apoptosis Detection Kit featuring fluorescein isothiocyanate (Cat. No. 40306ES20) was purchased from Shanghai YEASEN (Shanghai, China). DAPI (Cat. No. 28718-90-3) was obtained from Proteintech (Rosemont, IL, United States). Apoptosis was evaluated after drug treatment *in vivo*, following the manufacturer’s instructions.

The TUNEL assay was performed as described by Loo (20). Briefly, tissues were fixed in formaldehyde and permeabilized with Proteinase K to allow the penetration of TUNEL reaction reagents into the cell nucleus. After fixation and washing, the incorporation of biotinylated dUTP onto the 3′ ends of fragmented DNA was conducted in a reaction containing terminal deoxynucleotidyl transferase. The slides were mounted with 90% glycerol and visualized by fluorescence microscopy. The TUNEL stained slides were calculated by manual counting under a fluorescent microscope. The TUNEL-stained cells appeared green, while the other cell nuclei appeared blue. The apoptosis index (AI) was regarded as the number of TUNEL-positive cells/total number of cells × 100%.

### Immunohistochemistry

Immunohistochemistry (IHC) was performed as previously described (21). Briefly, paraffin-embedded xenografts or tissues were cut into 3-μm sections and mounted on slides, subjected to antigen retrieval in hot citrate buffer (pH = 7.4), then blocked in 10% normal goat serum. Subsequently, sections were incubated with primary antibodies against Ki-67 or proliferating cell nuclear antigen (Cat. Nos. 27309-1-AP and 10205-2-AP PCNA; Proteintech). The slides were incubated with goat anti-mouse/rabbit poly-horseradish peroxidase-conjugated secondary antibodies (Cat. No. PR30009; Proteintech). Nuclear Ki-67, as well as nuclear and cytoplasmic PCNA, stained red clay or brown. The PCNA slides were scored and analyzed using Image-Pro Plus software. Six 400X images were analyzed for each slide. The average integrated optical density was calculated as the ratio of the positive area to the total area. The Ki67 slides were analyzed using a microscope. Six 400X images were analyzed for each slide. The positivity cell rate was calculated as the ratio of the number of positive cells to the number of total cells.

### Statistical Analysis

Statistical analyses were performed using the SPSS software package (ver. 22.0; IBM, United States). All graphs were produced using Graph Pad Prism ver. 7.0 for Windows (Graph Pad Software Inc., United States). All experiments were performed in triplicate, with the means of those three independent experiments calculated. Data are presented as the means ± standard deviations (SDs) and were compared using Student’s t-test (two groups) or one-way ANOVA (multiple groups). A *p*-value < 0.05 was considered to indicate statistical significance.

## Results

### *In Vitro* Drug Sensitivities

Tumor samples from nine HNSCC patients were cultured *in vitro* at 37°C under 5% (v/v) CO_2_ (Table 1). The samples were labeled as Control, DMSO, anlotinib, sunitinib, apatinib, paclitaxel, and cisplatin. We used the MTT assay to assess tumor cell viability; anlotinib significantly inhibited cell viability (Figure 1A; Table 1). For all nine samples, anlotinib exhibited a greater inhibitory effect than did sunitinib and apatinib. The tumor inhibition rates were as follows: DMSO, 10.87 ± 6.58%; paclitaxel, 50.05 ± 11.33%; cisplatin, 41.88 ± 8.55%; anlotinib, 51.05 ± 13.74%; sunitinib, 30.03 ± 12.85%; and apatinib, 25.06 ± 16.37% (Figure 1B). Because drug inhibition rate >30% was regarded as an indicator of drug sensitivity, anlotinib treatment presumably resulted in significant tumor suppression *in vitro*.

**TABLE 1:** Drug inhibition of HNSCC tissue proliferation.

Sample number	Histological origin	Tumor inhibition rate (%)					
		DMSO	Paclitaxel	Cisplatin	Anlotinib	Sunitinib	Apatinib
No. 3	Oropharynx	5.11 ± 1.45	44.92 ± 1.80	42.05 ± 1.00	44.57 ± 0.76	27.56 ± 1.09	35.62 ± 0.90
No. 4	Oropharynx	9.46 ± 0.65	55.26 ± 0.64	44.62 ± 0.75	51.64 ± 0.72	17.98 ± 1.03	38.09 ± 0.71
No. 7	Larynx	5.00 ± 0.21	44.44 ± 0.06	36.76 ± 0.06	32.41 ± 0.43	21.38 ± 0.59	1.63 ± 0.50
No. 8	Larynx	18.78 ± 0.26	46.65 ± 0.37	40.85 ± 0.12	70.29 ± 0.10	16.39 ± 0.09	13.18 ± 0.15
No. 10	Hypopharynx	6.20 ± 0.41	49.66 ± 0.12	54.51 ± 0.10	68.97 ± 0.04	24.63 ± 0.04	13.69 ± 0.15
No. 12	Larynx	9.30 ± 0.72	39.02 ± 2.60	43.11 ± 0.41	44.26 ± 0.39	36.11 ± 0.53	21.57 ± 0.47
No. 15	Oropharynx	5.54 ± 0.28	37.37 ± 0.02	24.74 ± 0.15	31.51 ± 0.25	34.52 ± 0.13	28.16 ± 0.12
No. 17	Larynx	24.95 ± 0.27	77.3 ± 0.14	36.55 ± 0.22	64.83 ± 0.15	61.46 ± 0.21	59.31 ± 0.22
No. 19	Oropharynx	13.51 ± 0.07	55.78 ± 0.13	53.74 ± 0.22	51.01 ± 0.20	30.21 ± 0.10	14.28 ± 0.16

Absorbance (A) at 490 nm was used to calculate drug sensitivity as follows: tumor inhibition rate = (1—drug A/control A) × 100%; tumor inhibition rate ≥30% indicates drug sensitivity.

**FIGURE 1:** **(A)** Representative results: 7-days drug sensitivity of HNSCC tissues measured using the MTT assay. **(B)** Quantitative data from three independent experiments are shown in the right panels. *p < 0.05; **p < 0.01.

### Anti-Tumor Effects of Anlotinib *in vivo*

Given the *in vitro* data, nine PDXs (numbered as P0) were established. Three PDX models were selected and passaged to P3 by the same method, then used for *in vivo* experiments. Mice bearing the PDXs were treated with drugs for 21 days, at which time the tumor volume in the control groups reached 1,500 mm^3^. The mice were then sacrificed. No mouse lost more than 10% of its body weight during the experiment, and no abnormal behavior was noted. Anlotinib was significantly more inhibitory (TGI 79.02%) than cisplatin (TGI 40.57%) (Figure 2A). The tumor volume in the anlotinib group on day 21 did not differ significantly from the initial volume (Figure 2B). The tumors in the anlotinib group were smooth-surfaced (unlike the tumors in the other two groups).

**FIGURE 2:** Anti-tumor effects of anlotinib in the PDX model. **(A)** Representative tumor images after treatment. **(B)** Tumor volumes every 4 days. When the volume in the control group reached 1,500 mm^3^, all tumors were harvested.

### Anlotinib Inhibits Tumor Cell Proliferation

To evaluate the anti-tumor effects of anlotinib, the Ki-67 and PCNA indices of tumor sections were immunohistochemically evaluated. The Ki-67 and PCNA expression levels differed significantly among the three groups (Figure 3A). In the anlotinib group, the Ki-67 positive rates were 20.26 ± 1.60% for patient no. 8, 26.7 ± 4.47% for patient no. 10, and 25.13 ± 3.24% for patient no. 17; these were significantly lower than the rates in the control group (61.89 ± 4.44% for patient no. 08, 55.16 ± 6.17% for patient no. 10, and 55.85 ± 2.23% for patient no.17; *p* < 0.05) (Figure 3B). Similarly, compared to the control group, the PCNA-average integrated optical densities of 0.19 ± 0.01, 0.15 ± 0.01, and 0.10 ± 0.01 for patients no. 8, 10, and 17, respectively, were significantly lower than (*p* < 0.05) the corresponding figures in the control group (0.50 ± 0.01, 0.35 ± 0.01, and 0.21 ± 0.01) (Figure 3C). The Ki-67-positivity rates and PCNA-average integrated optical densities were lower in the anlotinib group than in the positive control group, suggesting that tumor growth was inhibited in HNSCC PDX mice; moreover, anlotinib significantly inhibited tumor cell proliferation.

**FIGURE 3:** **(A)** Representative image of immunohistochemical staining for Ki-67 and PCNA in mouse tumor tissues (scale bar: 20 µm). Nuclear Ki-67, as well as nuclear and cytoplasmic PCNA, are stained clay red or brown. Percentages of cells expressing Ki-67 **(B)** and PCNA average IOD **(C)** in the various groups (*, *p* < 0.05).

### Anlotinib Promotes HNSCC Tumor Cell Apoptosis

Hematoxylin-and-eosin staining of the HNSCC tumor tissues of three tumor-bearing mice showed that the extents of necrosis and apoptosis varied among the groups. Tumors actively proliferated in the control group, but less so in the positive control and anlotinib groups. Apoptosis was maximal in the anlotinib group, in which karyopyknosis, karyorrhexis, and apoptotic bodies were observed (Figure 4A). TUNEL assays were performed, with green fluorescence indicating apoptosis and nuclei fluorescing blue. The highest apoptosis levels were observed in the anlotinib group (Figure 4B) (patient no. 8: 27.03 ± 1.09%, no. 10: 28.69 ± 0.96%, and no. 17: 41.12 ± 1.21%; the control values were no. 8: 5.01 ± 0.63%, no. 10: 5.245 ± 0.33%, and no. 17: 9.69 ± 0.52%; and the positive control values were no. 8: 9.50 ± 0.58%, no. 10: 11.50 ± 0.71%, and no. 17: 9.94 ± 1.648%) (*p* < 0.05) (Figure 4C). Therefore, anlotinib promoted tumor cell apoptosis.

**FIGURE 4:** Anlotinib exerts anti-tumor effects by promoting apoptosis. **(A)** Hematoxylin-and-eosin staining of tissue from PDX no. 17. Active tumor proliferation was observed in the control group, less proliferation was observed in the cisplatin group, and apoptosis (as revealed by karyopyknosis and karyorrhexis) was observed in the anlotinib group. **(B)** Microscopic TUNEL fluorescence (cell numbers >100) (green fluorescence, positive cell signal; blue fluorescence, nuclear staining). **(C)** The signal was significantly higher in the anlotinib group (*, *p* < 0.05).

## Discussion

HNSCC treatment remains challenging, although a multidisciplinary approach improves outcomes and increases survival. Local and distant metastases are the most important prognostic factors (22); several studies have shown that the expression of angiogenic factors and their receptors are closely related to the development, metastasis, and prognosis of HNSCC. Identifying drugs that suppress tumor development and metastasis is both important and difficult. Anti-angiogenesis inhibitors reduce tumor blood supply, create a low-oxygen microenvironment, and improve the efficacy of chemotherapy (23). Anlotinib is a small molecule, newly developed, oral and multi-targeting tyrosine kinase inhibitor that targets VEGFR1, VEGFR2/KDR, VEGFR3, c-Kit, PDGFR-α, and the fibroblast growth factor receptors. Furthermore, it can inhibit both tumor angiogenesis and tumor cell proliferation (16, 24–26). Therefore, anlotinib anti-angiogenesis in combination with chemotherapy is a promising direction of research.

Although drugs targeting the vascular system effectively treat a variety of tumors, the therapeutic responses differ. Thus, selection of an appropriate drug is key in terms of personalized and precision medicine. Simple, individualized preclinical drug screening is important in this context. Most researchers of cancer biology use two- or three-dimensional models that have intrinsic limitations and may exhibit poor reproducibility. PDXs have been increasingly used for drug screening and evaluating drug resistance. PDXs retain tumor heterogeneity throughout implantation and *in vivo* culture. We subcutaneously implanted HNSCC tumor tissues into immunodeficient mice to establish PDXs for drug screening. Finally, nine PDXs (numbered as P0) were established. Three PDX models were selected and passaged to P3 by the same method, then used for *in vivo* experiments, because they were more efficient in developing tumors; moreover, their tumor sizes were similar. *In vitro*, anlotinib and paclitaxel suppressed tumors similarly. However, the individual results differed greatly. PDXs maintain the genetic characteristics of the parental tumors and recapitulate human tumor biology. They allow evaluation of the effects of different drugs in single patients and the effects of the same drug in different patients. Our average cisplatin tumor inhibition rate was 41.88 ± 8.55% *in vitro*, and the TGI was 40.57% *in vivo*. Thus, the *in vivo* and *in vitro* data were consistent. However, the anlotinib inhibition rates differed significantly *in vivo* and *in vitro*; the former rate was higher. Hence, when using PDXs, it is important to consider drug absorption and metabolism.

Previous studies found that the expression of VEGF, FGFR1–4, and their receptors markedly affected tumor aggressiveness and prognosis; however, little research on how this affects HNSCC has been published (27, 28). Angiogenesis is very important in terms of tumor growth and metastasis; accordingly, anti-angiogenic agents are major components of current tumor treatments (29, 30). We found that anlotinib exhibited a better anti-tumor effect than did cisplatin. The tumor volumes in the anlotinib group did not increase significantly from the initial volumes. This allows a new clinical strategy. It is essential to improve the prognosis of patients with advanced HNSCC.

Of the many vascular factors, VEGF and its receptor VEGFR play key roles in tumor angiogenesis. Binding of VEGF to the receptor triggers receptor phosphorylation and the activation of downstream signaling by STAT3, Akt, and Erk-1/2, followed by endothelial cell proliferation, migration, and tube and microvessel formation (31, 32). Anlotinib targets JAK2/STAT3/VEGFR signaling, and the inhibition of angiogenesis halts tumor proliferation and promotes apoptosis (16, 17, 33–35). Anlotinib is a potent tyrosine kinase inhibitor that inhibits VEGFR2 phosphorylation as well as that of PDGFRα/β, c-Kit, RET, Aurora-B, C-FMS, and the discoid region of DDR1 (14, 15). Although anlotinib binds to both VEGFRs and other targets, the drug is more selective for VEGF family members (especially VEGFR2 and VEGFR3) than is sunitinib. Anlotinib selectively inhibits VEGFR-dependent tumor cell proliferation, as described above. We confirmed that anlotinib suppressed HNSCCs *in vivo*, as revealed by the Ki-67 and PCNA immunohistochemical data. Compared to cisplatin (the positive control), anlotinib exhibited a greater inhibitory effect. Anlotinib also promoted tumor apoptosis.

Our results indicate the potential for anlotinib-sensitive HNSCC tumors. However, three PDX models were involved in *in vitro* experiments; other tumors may be resistant to anlotinib. More studies are needed to reveal the possible reasons. In addition, studies are needed to explore the mechanisms and determine the appropriate selection method to identify patients who may benefit from a treatment that includes anlotinib.

## Conclusion

We successfully established a PDX model of HNSCC. To our knowledge, this is the first study to show the role of anlotinib in HNSCC *in vivo*. Anlotinib exhibited good anti-tumor activity *in vitro* and *in vivo*, inhibiting cell proliferation and promoting apoptosis. These findings suggest that anlotinib could be used for the treatment of patients with HNSCC.

## Data Availability

The original contributions presented in the study are included in the article/Supplementary Material, further inquiries can be directed to the corresponding authors.
